# Anticancer and Free Radical Scavenging Competence of Zinc Oxide Nanoparticles Synthesized by Aqueous Leaf Extract of *Phyllanthus acidus*

This article has been retracted.

**DOI:** 10.1155/2022/9493816

**Published:** 2022-08-25

**Authors:** Arunachalam Chinnathambi, Sulaiman Ali Alharbi, Deepika Joshi, Haiter Lenin

**Affiliations:** ^1^Department of Botany and Microbiology, College of Science, King Khalid University, PO Box-2455, Riyadh 11451, Saudi Arabia; ^2^Department of Oral Biology, University of Louisville, Louisville, Kentucky, USA; ^3^Department of Mechanical Engineering, WOLLO University, Kombolcha Institute of Technology, Kombolcha, Ethiopia

## Abstract

The purpose of this study was aimed to investigate the zinc oxide nanoparticles (ZnONPs) synthesizing efficiency of aqueous leaf extract of *Phyllanthus acidus.* Furthermore, the antioxidant and anticancer activities of synthesized ZnONPs were also investigated through the in-vitro approach. The obtained results show that the aqueous extract of *P. acidus* can synthesize ZnONPs, as evidenced by a sharp absorbance peak at 375 nm. The Fourier transform infrared spectroscopy (FTIR) analysis confirmed that the aqueous extract contained significant numbers of functional groups, which were involved in reducing zinc nitrate into ZnONPs. Also, they participate in the capping and stabilization of synthesized ZnONPs and their size ranged from 27.14–35.74 nm with a spherical shape . The results obtained in ABTS radical scavenging activity 1, 1-diphenyl-2-picryl-hydroxyl (DPPH), hydrogen peroxide (H_2_O_2_), and 2,2′-Azino-Bis(3-ethylbenzene thiazoline-6-sulfonic acid) (ABTS) assays declared has excellent in-vitro radicals scavenging activity with reasonable IC_50_ values. Interestingly, these green synthesized ZnONPs have an excellent anticancer activity against human epidermoid carcinoma (Hep3) cell line in an in-vitro approach. These findings imply that an aqueous leaf extract of *P. acidus* can be used to synthesize pharmaceutically valuable ZnONPs. To consider such nanomaterials as potential therapeutic agents, optimization and in-vivo biomedical studies are required.

## 1. Introduction

Metal nanoparticles are gaining more attention in recent years among researchers to fabricate nanoparticles from various metals through different fabrication processes such as physical, chemical, and biological methods. Zinc oxide nanoparticles have a substantial degree of positive influence on biological applications compared to other noble metals such as silver, zirconium, cadmium, lead, copper, cobalt, aluminum, and gold [1, 2]. Since zinc is one of the essential trace elements required for essential metabolic activity and regular cell functions, its notable essential roles are catalytic, structural, and regulatory ions, and it contributes significantly to the immune system, apoptosis, homeostasis, and oxidative stress [3, 4]. The metallothioneins are a group of zinc-binding specialized proteins, and they protect the cells from stress and toxic conditions induced by toxic metals. During aging and degenerative disease conditions, these zinc elements rectify the immune defects, minimize infection relapse, and inhibit aging [5]. Hence, in this study, the oxide form of zinc nanoparticles has been focused on due to the excellent reactivity of zinc nanoparticles. Conventional physical and chemical methods can synthesize these nanoparticles. Nevertheless, these approaches require a more sophisticated laboratory setup, not an ecofriendly, complicated process that includes a separate capping and stabilization process. Hence, the biological process overcomes these issues and yields well-capped and stabilized nanoparticles. Plant biomass, microbes, and biologicals have been identified as suitable source materials for the environmentally friendly synthesis of nanoparticles [6]. Plant biomass is naturally available with rich genetic variability and contains significant biomolecules among these biological sources. The plant biomass contained various biomolecules such as proteins, coenzymes, phenolic compounds, vitamins, flavonoids, and so on; these biomolecules contain several functional groups such as hydroxyl, amines, and carbonyls, which interact with metal ions and reduce them as nanoparticles. These biomolecules also possess a significant role in the capping and stabilizing of synthesized nanoparticles [7]. Hence, in this study a pharmaceutically well-recognized *Phyllanthus acidus* plant has been used, especially the leaf extract of this plant has been focused. This is the very first report on the fabrication of zinc oxide nanoparticles from zinc acetate using *Phyllanthus acidus* aqueous leaf extract and the assessment of their antioxidant and anticancer potential in-vitro [8]. Other species of *Phyllanthus* namely *Phyllanthus Emblica* stem and seed powder extract have been reported as a potential to reduce, cap, and stabilize ZnONPs from zinc acetate/nitrate [9]. These plants contain a considerable number of pharmaceutically valuable phytochemicals such as alkaloids, flavonoids, tannin, saponins, phenols, and so on [10]. Globally, the peoples are either directly or indirectly suffered from excess accumulation of free radicals. It can worsen and contribute to a variety of chronic health problems, including cataracts, cancer, inflammatory, and cardiovascular diseases [11]. They could either donate or accept electrons from essential biomolecules and thus act as oxidants or reductants [12]. The most significant oxygen-containing free radicals, such as –OH, O^2-^, H_2_O_2_, ClO, NO, and peroxynitrite radicals, were discovered to be responsible factors in a variety of disease conditions [13]. These are extremely reactive species capable of damaging biologically important components such as DNA [14], proteins [15], carbohydrates [16], and lipids in the nucleus and cell membranes. Globally, cancer is a leading cause of death and accounting for almost 10 million demises in 2020. Cancer is the first or second major cause of mortality in 91 of 172 nations, and it ranks 3^rd^ or 4^th^ in another 22 nations. Cancer is the 2^nd^ and 4^th^ leading cause of adult mortality in both urban and rural India [17]. As per the author's knowledge, this is the first report about the anticancer and free radicals scavenging potential of ZnONPs synthesized by P. *acidus* extract. The nanoparticle synthesizing efficiency of this test plant has not been reported previously. Hence, this research was designed to evaluate the ZnONPs synthesizing potential of aqueous extract of P. acidus and their in-vitro antioxidant (DPPH, H2O2, and ABTS) and anticancer potential against Hep3 cell lines.

## 2. Materials and Methods

### 2.1. Plant Sample Collection and Processing

The fresh and disease-free *Phyllanthus acidus* leaf samples were collected from an agricultural land at Vadathorasalur, Kallakurichi district of Tamil Nadu, India. The collected plant leaves were washed with clean tap water to remove the dust and debris attached over the surface of the leaves and completely dehydrated under shadow conditions. Well, the dehydrated leaf sample was then pulverized using an electric pulverizer (AZ302-Creta Power, AATOMIZE, India). The powdered sample was stored in the refrigerator for further process.

### 2.2. Aqueous Extract Preparation

The fine powdered 20 g of the leaf sample was dissolved in 100 mL of distilled water in a 250 mL conical flask and kept in the water bath for 30 min at 50°C through the standard hot extraction method. The extract from the reaction mixture was then filtered using a Whatman number 1 filter paper, and the filtrate was concentrated by evaporating the water from the filtrate and subjected to nanoparticle synthesis.

### 2.3. Green Synthesis of ZnONPs

The condensed aqueous extract derived from the *P. acidus* leaf was used to synthesize the ZnONPs from zinc nitrate to assess their efficiency following the typical protocol. In brief, about 20 mL of the condensed aqueous leaf extract was mixed with 80 mL of freshly prepared 0.5 M zinc nitrate solution in a 250 mL conical flask. The reaction mixer containing a conical flask was incubated at 70°C for 48 h in a shaking incubator. After incubation, the obtained pale color precipitate was centrifuged at 3000 rpm for 25 min and the pellet was washed with Milli Q water and then dried in a hot air oven (50°C for 20 min). The aqueous leaf extract of *P. acidus* has excellent potential to reduce the zinc nitrate into zinc oxide nanoparticles (ZnONPs); it was initially screened by noticing a visible color alteration in the reaction mixer during the reduction time (i.e., synthesis) as yellowish-white residue. It indicates the reduction of zinc nitrate into nanoparticles. The dried particles were subjected to standard characterization techniques to determine the quality of the synthesized nanoparticles.

### 2.4. Characterization of Synthesized ZnONPs

#### 2.4.1. UV-Visible Spectral Analysis

The *P. acidus* aqueous leaf extracts synthesized ZnONPs were subjected to a UV-visible spectrophotometer (UV-vis spec. 2450, Shimadzu) analysis to confirm the presence of ZnONPs by scanning the sample ranging from 300 to 600 nm as per the standard operating protocol.

#### 2.4.2. Fourier-Transform Infrared (FTIR) Study

The standard FTIR analysis protocol was performed to investigate the functional groups belonging to the bioactive components present in the aqueous extract, which involved the reduction, capping, and stabilization potential of ZnONPs. The FTIR -1000, Perkin Elmer, (USA) model was used to investigate the functional groups involved in the synthesis process by scanning the sample with the spectral range of 4000–400 cm^−1^ with the resolution of 4 cm^−1^.

#### 2.4.3. Microscopic Structural Properties of ZnONPs

The morphological characteristics such as shape, size, and alignment form either agglomerated or uniformly or individually distributed form of aqueous leaf extract of *P. acidus* synthesized ZnONPs were investigated by scanning electron microscopy (SEM) and transmission electron microscopy (TEM). The standard operating protocols were followed for each microscopic observation using SEM (Mx 63 and Mx63 L Olympus) and TEM (Jem-1400Flash, Jeol).

### 2.5. Free Radicals Scavenging Assays

#### 2.5.1. 1, 1-Diphenyl-2-Picryl-Hydrazyl Radical Scavenging Activity

The DPPH (1, 1-diphenyl-2-picryl-hydrazyl) is one of the most essential free radicals, which is subjected to determine the free radicals scavenging competence of suspected test antioxidant molecules. The standard in-vitro assay protocol was followed to investigate the radicals scavenging potential of ZnONPs. In brief, 0.8 mL of 0.1 mM of DPPH was mixed with 1.2 mL of different concentrations of 50–250 µg mL^−1^ of aqueous leaf extract synthesized ZnONPs and kept under dark conditions for 30 min. Ascorbic acid was used as a positive control. Subsequently, the color change was observed and the absorbance of these tests and positive control were read at 517 nm using a UV-visible spectrophotometer (UV-vis spec. 2450, Shimadzu). The standard antioxidant percentage and IC_50_ value for the test and positive control were calculated using the standard formula.

#### 2.5.2. Hydrogen Peroxide (H_2_O_2_) and ABTS Scavenging Assays

The H_2_O_2_ radicals scavenging efficiency of green synthesized ZnONPs was studied by following the typical methodology. About 1.2 mL of various concentrations of 50–250 *µ*g mL^−1^ of ZnONPs were blended with 0.8 mL of freshly prepared 40 mM H_2_O_2_ solution respectively. Similar concentrations of ascorbic acid were used as a positive control. These reaction blends were then incubated at room temperature for 20 min, and the absorbance of positive and tests was read at 230 nm using a UV-visible spectrophotometer. The standard formula was used to calculate the scavenging percentage and IC_50_ values of test and positive control.

ABTS (2,2′-azino-bis (3-ethylbenzothiazoline-6-sulfonic acid)) is one of the most significant scavenging assays to determine the antioxidant efficiency of test antioxidant molecules. The standard ABTS assay methodology was followed to determine the antioxidant efficiency of various concentrations of *P. acidus* aqueous leaf extracts synthesized ZnONPs. In brief, about 980 *μ*L of day-old ABTS reagent (contained 7.0 mM of ABTS and 14.7 mM of ammonium peroxodisulphate) was mixed with 20 *μ*L of various concentrations of (50–250 *µ*g mL^−1^) of ZnONPs and kept at room temperature for 10 min under darkness. A similar dosage of ascorbic acid was used as a positive control, and the absorbance of this positive test were read at 734 nm through a UV-visible spectrophotometer. The scavenging percentage and the IC_50_ value were calculated using the standard formula.

### 2.6. Cytotoxicity Assay

The anticancer activity of ZnONPs synthesized by aqueous leaf extract of *P. acidus* was studied by using the 3-(4, 5-dimethylthiazol-2-yl)-2, 5-diphenyltetrazolium bromide (MTT) assay on Hep3 cell line (human epidermoid carcinoma #3 cells) through an in-vitro approach using the typical experimental procedure. In brief, well-maintained Hep3 cell line (approximately 5000 cell mL^−1^ concentration) was seeded on 96 well plates in triplicates and treated with 50 and 100 *μ*g mL^−1^ dosages of ZnONPs added to each well. Subsequently, about 60 *μ*M of curcumin was used as a positive control and 0.5% of dimethyl sulfoxide (DMSO) was used as a negative control. Then, the plates were incubated at 37°C for 24 h in a 5% CO_2_ chamber and the cells containing wells were rinsed with phosphate-buffered saline (PBS) solution. Subsequently, 100 *μ*L of freshly prepared MTT solution was added to each well and incubated again at 37°C for 4 h. About 100 *μ*L of the DMSO reagent was added to each well after the incubation and placed in a shaker for few minutes to confirm the complete dissolving of MTT crystals. Then, the absorbance value of each well was recorded at 545 nm. The cytotoxicity percentage and IC_50_ values of the test and positive control were determined by applying the standard formula.

## 3. Results and Discussion

### 3.1. Green Fabrication of ZnONPs

The results obtained from this study indicated that the aqueous leaf extract contains a significant quantity of metal-reducing bioactive components in the form of phytochemicals, since some proteins, coenzymes mediated product, total phenolic compounds, flavonoids, and so on can reduce the metals into nanosized particles. This result was exactly correlated with the findings of ZnONPs synthesized by aqueous leaf extract of *Devera tortuosa* was reported to develop a yellowish white precipitate and considered an indication of zinc nitrate reduction into nanoparticles [18]. The UV-visible spectrum analysis results revealed that the major absorption peak for ZnONPs synthesized by aqueous leaf extract of *P. acidus* was found at 375 nm (Figure 1).

Several reports stated that the range of absorption peak for ZnONPs exists between 330–460 nm. This wide range of absorbance of ZnNPs might be directly related to the types of reducing agents used, reaction time, and amount of zinc nitrate/acetate subjected to the nanoparticle's synthesis [19]. The natural bandgap absorption of ZnO due to electron transfers from the valence to the conduction band could account for this absorption peak [20]. The peak obtained in this study was completely correlated with the absorbance peak of ZnONPs (374 nm) synthesized by whole plant aqueous extract of *D*. *tortuosa* [18].

### 3.2. Fourier-Transform Infrared Analysis

The functional groups, involved in the reduction, capping, and stabilization of ZnONPs, were investigated by FTIR analysis. The obtained FTIR results showed that the 12 predominant peaks (3407, 2585, 2108, 1645, 1586, 1549, 1385, 1258, 1090, 933, 835, and 517 cm^−1^) corresponded to various significant functional groups (Figure 2) of different bioactive components belong to several phytochemicals which capped over the surface of ZnONPs.

The peak obtained at 3407 cm^−1^ was related to stretched hydrogen bonds, 2585 cm^−1^ assigned to C–H stretching vibrations of the alkenyl group, 2108 cm^−1^ might be related to -C^_^C- stretching vibrations, 1645 cm^−1^ assigned to C=O stretching vibrations, 1586 cm^−1^ could be assigned to C=C/amine–NH stretching vibrations corresponding to aromatic compound, 1549 cm^−1^ assigned to COO- symmetric stretching vibrations, 1385 and 1258 cm^−1^ were assigned to C–H stretching vibrations, 1090 cm^−1^ could be related to the symmetric stretching vibration of amine group, 933 and 835 cm^−1^ were assigned to symmetric stretching vibrations of C–N corresponding to an amine, and 517 cm^−1^ could be assigned to stretching vibration related to ZnO (Figure 2).

The overall symmetric and asymmetric stretching vibrations bonds suggested hydrogen bonds, carboxyl, amine, and alkenyl groups. These functional groups were corresponding to various most significant bioactive components belonging to phytochemicals such as phenols, flavonoids, tannins, saponins, and so on can be involved in the reduction, capping, and stabilization. Hence, these molecules can reduce the zinc ions to zinc nanoparticles as Zn^2+^ to Zn^+1^ to Zn^0^ by donating the electrons from the extract [21]. The plant that contains more polyphenolic components can enhance the reduction of zinc nitrate to zinc oxide and stabilize the synthesized ZnONPs [22]. Furthermore, the obtained peaks assigned to various functional groups correlated to the previously published literature.

### 3.3. Scanning Electron Microscopy (SEM) and Transmission Electron Microscopy (TEM) Analyses

SEM and TEM analyses investigated the morphological appearance and size of ZnONPs synthesized by aqueous leaf extract of *P. acidus.* The obtained microscopic images revealed that the size of the ZnONPs ranged from 27.14–35.74 nm and was spherical in shape with an aggregated form and uniform distribution (Figures 3(a) and 3(b)).

These morphological results were correlated with the ZnONPs synthesized from *Sambucus ebulus* that ranged from 25–30 nm and mixed morphological appearance was reported as spherical and hexagonal shapes [23]. A similar pattern of morphological appearance has been reported in ZnONPs synthesized from the *Rubus fairholmianus* root extract showed the aggregated form of spherical-shaped nanoparticles with an average size of 11.34 nm [24]. The *Acantholimon serotinum* extracts mediated ZnONPs were reported as irregular spherical with a size ranging from 20–80 nm [25].

### 3.4. Antioxidant Activity Analysis

#### 3.4.1. 2,2-Diphenyl-1-Picrylhydrazyl Assay

The dose-dependent radicals scavenging activity was noted in the DPPH assay since the increased concentration showed maximum DPPH radical scavenging activities as 87.82% at the concentration of 250 *μ*g mL^−1^ concentration of green synthesized ZnONPs (Figure 4). Interestingly, this percentage was almost parallel to the positive control ascorbic acid scavenging activity (92.65%) and obtained scavenging percentage of ZnONPs was statistically significant at *P* < 0.03 to *P* < 0.05 (Figure 4).

IC_50_ values for ZnONPs and ascorbic acid were calculated as 126.90 and 112.61 *μ*g mL^−1^, respectively (Figure 4). A dose-dependent DPPH radicals scavenging activity was also reported in ZnONPs synthesized from the aqueous root extract of Scutellaria baicalensis and reported about 56.11% of DPPH radical scavenging at 1000 *μ*g mL^−1^ [26]. A similar range of DPPH radicals scavenging activity was reported in ZnONPs synthesized from the crude extract of *Turbinaria conoides*, it showed 69.4% DPPH radicals scavenging activity at 250 *μ*g mL^−1^ concentrations, and their IC_50_ value was reported as 157 *μ*g mL^−1^ [27]. These results suggest that the synthesized ZnONPs capped with significant functional groups can potentially reduce the 2,2-diphenyl-1-picrylhydrazyl into a yellowish diphenyl picrylhydrazine compound [23].

#### 3.4.2. Hydrogen Peroxide (H_2_O_2_) Scavenging Assay

The aqueous leaf extract synthesized ZnONPs have excellent H_2_O_2_ radicals scavenging activity in dose-dependent manner. The percentage of radicals scavenging activity was found as in the range of 47.18 to 84.23% at the concentrations of 50 to 250 *μ*g mL^−1^ concentrations of ZnONPs, and these almost resembled the radicals scavenging activity of ascorbic acid (55.21 to 87.89% for 50 to 250 *μ*g mL^−1^ concentrations). Furthermore, the obtained values were statistically significant at *P* < 0.03 to *P* < 0.05 (Figure 5).

The IC_50_ values for ZnONPs and ascorbic acid were estimated as 128.53 and 117.92 *μ*g mL^−1^, respectively. The ZnONPs synthesized from the crude extract of *Turbinaria conoides* have an excellent antioxidant activity on H_2_O_2_ at 51% at the concentration of 250 *μ*g mL^−1,^ and their IC_50_ value was determined as 236 *μ*g mL^−1^ [27]. Another report stated that the ZnONPs synthesized from *Sambucus ebulus* have a considerable level of H_2_O_2_ radicals scavenging activity with a very reasonable quantity of nanoparticles. According to this, the IC_50_ value of ZnONPs mediated from *S. ebulus* was found as 43 *μ*g mL^−1^ [23]. Another report stated that the *Albizia lebbeck* bark extract synthesized ZnONPs showed a significant level of H_2_O_2_ radicals scavenging activity. The IC_50_ value was reported as 60.0 *μ*g mL^−1^ [28].

#### 3.4.3. 2,2′-Azino-Bis(3-Ethylbenzothiazoline-6-Sulfonic Acid) (ABTS) Scavenging Assay

The ABTS radicals scavenging assay revealed that the ZnONPs synthesized by aqueous leaf extract of *P. acidus* have the radicals scavenging potential in a short duration of time in a dose-dependent manner. The ABTS radicals scavenging percentage was found as 87.82 to 92.65% for the concentration of 50 to 250 *μ*g mL^−1^, respectively. These percentages were close to the positive control radical scavenging activities of 57.89 to 92.65% at the concentration of 50 to 250 *μ*g mL^−1^, respectively, (Figure 6).

The IC_50_ values for ZnONPs and ascorbic acid were calculated as 127.55 and 113.12 *μ*g mL^−1^, respectively (Figure 6). The obtained values were statistically significant at *P* < 0.03 to *P* < 0.05. This result was comparable with the ABTS scavenging potential of ZnONPs synthesized from the aqueous root extract of *Sphagneticola trilobata* was reported as 86.88% at the concentration of 50 *μ*M and their IC_50_ value was found as 41.76 *μ*g mL^−1^ [29]. Similarly, another report stated that the aqueous fruit extracts of *Myristica fragrans* synthesized ZnONPs have 82.12% ABTS radicals scavenging activity at the concentration of 400 *μ*g mL^−1^ [30]. About 89% of ABTS radicals scavenging activity was found at 2800 *μ*g mL^−1^ concentration of ZnONPs synthesized from photosynthetic green algae *Sargassum muticum* extract [31].

### 3.5. *In-Vitro* Anticancer Activities

The ZnONPs synthesized by aqueous leaf extract of *P. acidus* has a considerable level of *in-vitro* anticancer activities against human epidermoid carcinoma (Hep3) cell lines. It was directly related to the dose-dependent manner. The anticancer activity percentage was calculated as ranging from 57.12 to 92.39% at the concentrations of 50 and 100 *µ*g mL^−1^ respectively (Figure 7), and it was almost comparable to the curcumin at 76.43 and 97.41% at the same concentration. Furthermore, the IC_50_ value of ZnONPs was found as 51.70 *µ*g mL^−1^ and this value was close to the IC_50_ value (46.08 *µ*g mL^−1^) of positive control curcumin (Figure 7). The ZnONPs synthesized from aqueous leaf extract of *Saponaria officinalis* reported that the IC_50_ value was 26.3 *μ*g mL^−1^, and 60.08 *μ*g mL^−1^ for HFF MDA-MB-231 cell lines [32]. A dose-dependent anti-breast cancer activity was reported for root extract of *Withania somnifera* synthesized ZnONPs on the MCF-7 cell lines and IC_50_ value was reported as 13.65 *μ*g mL^−1^ [33].

Similarly, the aqueous root extract of *Gracilaria edulis* synthesized ZnONPs showed a significant dose-dependent *in-vitro* anticancer activity against SiHa cells, and the IC_50_ value was found as 35 ± 0.03 *μ*g mL^−1^. The possible mechanisms involved in the anticancer activity of ZnO NPs on cancerous cells were reported as it can increase the accumulation of intracellular ROS and stimulate the cell to face the apoptosis process. The ZnONPs also induce mitochondrial damage and oxidative stress in cancer cells. The mitochondria are the most vital organelles required to regulate the signal transduction process, maintain the steady state level of apoptosis in mammalian cells, and control the cellular energy metabolism mechanisms in cancerous and normal cells. Thus, once the ZnONPs enter the cancerous cells, it causes damage to mitochondria and leads to cancer cell death.

## 4. Conclusion

*P. acidus* aqueous leaf extract contains significant amounts of the most efficient functional groups involved in the reduction of zinc nitrate to ZnONPs. In this study, color changes and a sharp absorbance peak at 375 nm, which corresponded to ZnONPs, were observed. Peaks in the FTIR analysis revealed the functional groups involved in the synthesis of these ZnONPs. They represented the number of functional groups that were found in various bioactive molecules. The green synthesized ZnONPs ranged in size from 27.14 to 35.74 nm and had a spherical shape. In-vitro antioxidant activity of these ZnONPs was demonstrated by DPPH, H_2_O_2_, and ABTS radical scavenging assays. Furthermore, these ZnONPs have a potent anticancer activity against the Hep3 cell line in vitro. These findings imply that P. *acidus* aqueous leaf extract can be used to synthesize valuable biomedical ZnONPs. As a result, further research into fabrication optimization and in-vivo analysis need to be done to ensure the pharmaceutical applications of ZnONPs.

## Figures and Tables

**Figure 1:** UV-visible spectrum analysis of ZnONPs synthesized by aqueous leaf extract of *P. acidus.*

**Figure 2:** FTIR spectra of *P. acidus* aqueous leaf extract synthesized ZnONPs.

**Figure 3:** Morphological analysis of green synthesized ZnONPs. (a) SEM analysis (b) TEM analysis.

**Figure 4:** DPPH radicals scavenging activity of ZnONPs. The mentioned values are the mean and standard error of triplicates. ^*∗*^ indicates a statistical significance at *P* < 0.03; ^∗∗^ indicates a statistical significance at *P* < 0.05.

**Figure 5:** H_2_O_2_ radicals scavenging activities of ZnONPs. The mentioned values are the mean and standard error of triplicates. ^*∗*^ indicates a statistical significance at *P* < 0.03; ^∗∗^ indicates a statistical significance at *P* < 0.05.

**Figure 6:** ABTS radicals scavenging activities of ZnONPs. The mentioned values are the mean and standard error of triplicates. ^*∗*^ indicates a statistical significance at *P* < 0.03; ^∗∗^ indicates a statistical significance at *P* < 0.05.

**Figure 7:** *In-vitro* anticancer activity of ZnONPs against Hep3 cell line. The mentioned values are the mean and standard error of triplicates. ^*∗*^ indicates a statistical significance at *P* < 0.03, ^∗∗^ indicates a statistical significance at *P* < 0.05.

## Data Availability

The data that support the findings of this study are available on request from the corresponding author.
